# Application of Motion Effect Evaluation Algorithm Based on Random Forest

This article has been retracted.

**DOI:** 10.1155/2022/2039423

**Published:** 2022-10-06

**Authors:** Jin Dong, Dengxiao Dong

**Affiliations:** Institute of Physical Education, Shanxi University, Taiyuan, Shanxi 030006, China

## Abstract

The development of big data technology makes the feature selection technology gradually perfect. The advantages of different feature selection technologies are different. Among them, random forest algorithm belongs to integrated feature selection algorithm. Integrated processing of classification results can screen out the most representative feature impact. Based on this background and random forest algorithm, this paper analyzes the evaluation of motion effect. After the measurement, this paper obtains the body data before and after the training. After the calculation, the change data of the body index are determined. The random forest feature selection method is used as the carrier to determine the corresponding index attribute set. In the process of data set input, the corresponding whole input data set is formed through data classification. The completion of training, through the comparative experiment, is conducive to clear the degree of influence of physical indicators and then complete the exercise effect evaluation. The research shows that the random forest algorithm has significant advantages in the evaluation of sports effect and can effectively improve the accuracy of classification.

## 1. Introduction

At present, motion effect evaluation involves multiple disciplines and is the focus of the current industry. There are relatively many types of algorithms, including linear discrimination, logistic regression analysis, and random forest. The application in evaluation is relatively common. The algorithm has a high degree of maturity. After application, it can effectively improve the accuracy of calculation results and supports a large number of variable processing and high-dimensional data processing. During the application process, it is conducive to promoting data balance and reducing errors appeared, with many advantages. By using the random forest algorithm to complete the exercise effect evaluation, it can effectively ensure the accuracy of exercise effect evaluation and provide a basis for the development of clinical-related industry research work [1].

With the rapid development of the Internet, intellectual property, and other information technology, information in many places like to gather. For example, in June 2019, Google received 6,049 billion visits and YouTube 2,431 billion. Home sites like Baidu reached 977 million, while other sites like Tencent and Sogou also reached more than 100 million. By January 2020, the number of social network users worldwide will reach 3.8 billion. Such a large stream of access should create all kinds of data networks. This shows that big data play an important role in national development, and the development and education of big data are an important part of modern needs and the focus on all segments of the community [2]. Sports data are an important part of big data resources. The mining and analysis of sports data can effectively understand the impact of sports on the human body and the efficacy of sports. Existing sports data only focus on extracting and creating key features of sports data and providing them with key features that use statistical methods to identify sports information. However, with the rapid improvement of data mining and training technology, it is not possible to delete sports data using statistical data alone [3].

## 2. Literature Review

### 2.1. Random Forest Algorithm

It is very important to understand the integration of training technology and data mining technology to maximize the use of training technology and analyze sports data and provide suggestions for the promotion and popularization of sports. The research on sports effect evaluation is to use sports physique data for data mining. This paper mainly uses the feature selection algorithm to carry out the effect evaluation research. The main method is to define the research problem as a classification problem and select useful features in the classification process to do the later research, and the research flow is shown in Figure 1.

Random forest algorithm is a classifier, which further extends the basic function of the decision tree algorithm and randomly forms multiple independent decision trees for data training and prediction. It is an extended variant of the Bagging algorithm and decision tree algorithm, and an integrated model. He creates multiple trees decided by random sampling a pattern and selecting items from them and finally votes on the results of all the trees decided to be the final result. It is thought that insufficient memory is a collection of uncut trees or tree regression, and the design team used the model of the training materials to select different products in the induction tree to write and make assumptions.  Figure 2 shows a diagram of the bag product algorithm.

Ma et al. used the random forest algorithm to study the factors affecting the success rate of P2P online lending, and they compared the prediction ability of the random forest algorithm with algorithms such as decision trees and Bayesian and artificial neural networks and obtained a random the forest algorithm has higher prediction accuracy. Using random forest to analyze the CSI 300 index and screen high-quality stocks, the random forest algorithm can be well combined with the stock market to achieve accurate classification [5]. See Figure 3.

It can be seen from the above that the random forest algorithm has many improvement ways and a wide range of application fields, and it has its unique advantages compared with other algorithms in data classification and prediction. Therefore, random forest is a relatively mature and excellent machine learning algorithm in machine learning [6].

### 2.2. Overview of Sports Algorithms

The study of the effects of sports is the study of the effects of sports on the human body. The main goal of the study is to understand the relationship between sports and body shape effects based on big data and to understand the development of sports technology. Abroad, the research in this field is extensive, and the research results are abundant, especially in the United States and Japan. In the middle of the nineteenth century, Eastham et al.analyzed the influence of body functions by testing and studying students. Later, the United States opened the door to the study of physical fitness, and people began to pay a lot of attention to the test and study of human body function. With the passing of time, the United States gradually improved the relevant physical experiments, began to establish and develop different physical measurement projects, studied the individual's reaction power, explosive power, and other physical qualities, and explored and studied the indicators affecting the body function, such as flexibility, endurance, muscle strength, and other body composition indicators [7].

In 1979, the State Sports Commission, together with the Ministry of Education and the Ministry of Health, began to investigate the physical fitness of children and adolescents through statistical analysis of physical fitness monitoring results. This is the first time to comprehensively grasp the physical health status of children and adolescents in my country and has obtained important and valuable research results, which have attracted widespread attention from the society. At present, many domestic research institutes and colleges and universities have carried out theoretical and applied research in this field. For the research on physical fitness monitoring indicators of Chinese adults, domestic body shape indicators are more than in foreign countries. China uses pulse, blood pressure, vital capacity, step test, and other functional test indicators to evaluate research. Foreign countries generally choose brisk walking and step test. There are few quantitative studies [8, 9]. On the other hand, according to statistics, there is no good public database for sports data mining, which also brings difficulties to relevant research. As sports and information technology develops, some scholars have suggested the use of mathematical and computer devices to study sports data, and study the usefulness of sports information. Reliance on statistics is the most widely used way to achieve this goal.  Figure 4 shows the changes in the adult male body mass index between 2014 and 2010.

## 3. Database Establishment

### 3.1. Data Acquisition

In order to study the evaluation method of sports effect, the research team organized a number of subjects to conduct four types of sports training, namely wrestling, foot competition, skill, and modern school sports for a period of time, and observed more than 40 representatives of the subjects after training. Changes in indicators, such as body shape, physical function, and physical quality, and the changes in physical indicators are used as features to represent the observation object. First, the team divided sports into five categories: wrestling, skill, competitive foot, modern school sport, and no sport [10]. The establishment of no sports, not special sports test, is to reflect the impact of different sports on the body indicators. 785 students were tested in five sports categories, divided into five groups that played different sports. Before the exercise, the team measured the physical indicators of each group and recorded the data as *p*_0_. During the physical training, each group will have corresponding training for three months under the guidance of special personnel. The exercise cycle is three times a week, with seven minutes of preparation, 30 minutes of exercise, and three minutes of finishing. The index data at the end of the training were denoted as *P*. The team used a height and weight tester to measure height and weight, and a sitting height tester to measure sitting height. More than 40 physical indexes such as basic heart rate, cardiac work index, selective response time, and grip strength were measured by electronic human voice metronome, electronic sphygmomanometer, spirometer, handgrip meter, and reaction time tester [11].

### 3.2. Data Preprocessing

Predocumentation procedures include the removal of special objects, the resolution of inefficiencies, the coding behavior, and the data structure. Removing unique attributes refers to removing those attributes that cannot describe the distribution law of samples, such as some common ID attributes. Dealing with missing values is to deal with incomplete or missing data in data. Generally, there are three methods for missing value processing methods: completion, deletion, and direct use. Among them, the method of deleting attributes with missing values is suitable for very few attributes. Value contains a large number of missing values, to obtain more effective results [12]. The common missing value completion methods include mean value interpolation, mode interpolation, and intermediate value interpolation. When the feature is numerical data that can be calculated, attribute coding can be carried out. Attribute coding is usually characterized by dualism, that is, setting thresholds to divide numeric attribute values into 1 and 0 and convert them into Boolean types. Data normalization scales a column of data attributes to a state with a mean of 0 and a variance of 1. Data normalization uses formulas to normalize all data attributes into the same interval. In this process, we mainly did the following parts of the pretreatment. First, the unique attribute was removed. The unique attribute here was the ID attribute in the index data set, such as the “name” attribute in the obtained data [13]. These attributes could not describe the distribution rule of the sample, so we simply deleted the unique attribute. Second, for a small number of missing values in the processed data set, the method of mean interpolation is used to complete the missing values of the data; for example, the missing values of some male students in the same category are interpolated with the mean values of other male students in the same grade [14]. Third, the attribute data we deal with are all numerical data, which can carry out feature coding. Therefore, the characteristics are coded, and some attributes are converted into Boolean attributes, such as “one-minute tennis ball toss.” We take advantage of the data difference before and after training and set 0 as the cut-off point. The positive attribute value is 1, and the negative attribute value is 0. Finally, the data are normalized. Data normalization is to scale the attributes of the sample to a specified range. This paper mainly normalized the data difference before and after the test to between 0 and 1 [15].

The index data of the research object before and after training represent $p_{0}=\left\{\underset{Nx32}{\left.\overset{\mathrm{ij}}{x}\right\}}\right.$ and $p_{1}=\left\{\underset{\mathrm{nX}32}{\left.\overset{\mathrm{ij}}{y}\right\}}\right.$*N* is the number of people tested, *P*_0_ is the index data after three months of training, and the change of the index before and after training is expressed as

(1) $$\begin{array}{c} P=\frac{\left|\left(p_{1}-p_{0}\right)\right|}{\left.p_{0}\right|}\text{.} \end{array}$$

### 3.3. Database Establishment

In this essay, index change data were calculated by measuring index data before and after training. After data normalization and other data pretreatment steps, a total of 785 index change data with category markers were obtained. Further, the research team cooperated with sports experts to obtain ranking annotation of the real impact degree of sports data on indicators. According to experience, *z* voters voted in order based on the influence of such sports on indicators and summed the voting results to obtain the importance of physical indicators (Impact):

(2) $$\begin{array}{c} {Impact}_{c}\left(a_{p}\right)=m=\overset{Ζ}{\underset{m=1}{\sum }}vote\left(m{,a}_{p}\right)\text{,} \end{array}$$

where *I*mpact_*c*_(*a*_*p*_) represents the importance of type *C* exercise to item *P*, *m* represents voter *m*, and *Z* represents the total number of voters. In the experiment, there were 5 voters, *z* = 5. Database category vector *C*={*C*_1_*C*_2_, *C*_3_, *C*_4_, *C*_5_}, where *C*_1_ to *C*_5_ represent wrestling class, competitive foot class, skill class, modern school sports class, and nonsports class, respectively.

Experts were given four types of sports and were invited to vote on the influence degree of each type of sports on 32 indicators according to their experience. Then, the expert voting results were cumulative, and the sequence of top 10 indicators with significant influence of the four types of sports was obtained by ranking them from high to low. Finally, the ground-truth ranking of the real influence degree of sports on physical indicators is constructed, and the database of the influence degree of sports on physical indicators is constructed by combining the labeled information with the obtained data [16].

## 4. Research and Application of Motion Effect Evaluation Algorithm of Random Forest

### 4.1. Building a Decision Tree

A random forest is a classifier that contains multiple decision trees. Therefore, with the random forest method, the first step is to build a decision tree. A decision tree is a basic classifier that generally divides features into two categories [17]. The trees decide the operations recursively until the data set is divided into two categories. In this process, we use information gain to test whether the features produce nodes.

This article takes sports as an example to complete the construction of decision tree.  Figure 5 shows the relationship between entropy and probability in binomial distribution.

In the database, you can select indicators of physical activity's impact on the body, namely “characteristics,” database attribute set = A = {*a*_1_,*a*_2_, ..., *a*_P_}. Among them, database *P* contains 32 dimensional attributes, each of which has multiple possible values. In this paper, nonsports sports (marked as *C*_5_) and competitive foot sports (marked as *C*_2_) are taken as sample sets, with a total of 32 indicators. According to the characteristics of indicators, there are *V* possibilities, and the value is {*a*_1_, *a*^2^, ..., *a*^*v*^}. If the indicator is divided into training set *D*, *V* branches exist, and nodes are generated. Among them, the vth branch represents the sample that takes av on the feature α, information entropy of D is denoted as Dv.Ent(D), and the calculation formula is as follows:

(3) $$\begin{array}{c} Ent\left(D\right)=-\overset{\left|y\right|}{\underset{q=1}{\sum }}P_{q}\log_{2}P_{q}\text{,} \end{array}$$

where *P*_*q*_ = (*q* = 1,2, ..., |*y*|) represents the proportion of class *q* samples in the current sample set *D*. Considering that different branch nodes contain different number of samples, the weight |*D*^*v*^|/|*D*| is assigned to branch nodes in this essay, so the information gain obtained by attribute *a* on sample set *D* can be calculated.

(4) $$\begin{array}{c} Gain\left(D,a\right)=Ent\left(D\right)-\overset{V}{\underset{v=1}{\sum }}\frac{\left|D^{v}\right|}{\left|D\right|}Ent\left(D^{v}\right)\text{.} \end{array}$$

### 4.2. Evaluation Algorithm

Each time a decision tree is made, data are provided from the sample to indicate the decision tree, and unused data are used to measure the effectiveness of the decision tree. For each decision tree, select the corresponding out-of-bag (OOB) data to calculate the prediction error rate, randomly add noise interference to the feature *X* of all samples of the out-of-bag data, and calculate the out-of-bag data error again. Assuming that there are *N* trees in the forest, the average of the error values of the *N* trees is calculated to represent the importance of the feature *X*. Add random noise to study changes in prediction error rates and select important features.  Figure 6 is a branch graph of the root node based on the maximum ratio in the case of two types of multivalues, and Figure 7 is a branch graph of the root node in the case of multivalued attribute values.

Each time a certain proportion of features are removed, the information gain is used for attribute selection, and a new attribute set *a*_*x*_ is obtained.

(5) $$\begin{array}{c} a_{x}=\underset{a\in A}{argmax}Gain\left(D,a\right)\text{.} \end{array}$$

In this article, by taking competitive multiple sports as sample sets, the sports effect evaluation algorithm is constructed to obtain the impact degree of competitive foot sports on physical indicators, so as to evaluate the sports effect. When studying other types of sports, the above algorithm is also used to obtain the index attribute set that all kinds of folk sports have a great influence on the body index. The influence of corresponding sports on physical indexes was analyzed and inferred through the attribute set of indexes with great influence obtained from the study. The influence degree of different sports on physical indicators obtained by the algorithm was compared and evaluated with ground truth, and the accuracy of the algorithm was verified by the evaluation method.  Figure 8 shows the flow of the algorithm in this chapter.

## 5. Experimental Results and Discussion

### 5.1. Experimental Settings and Standards

The data used in the experiment are from the sports database SED. The method in this chapter is tested on the SED database, which is set as training set and test set with a ratio of 4 : 1. This paper mainly studies the influence of the four types of sports on the changes in the body's indicators. The data obtained from the sports experiment are used as the positive category, and the no sports data are used as the negative category, and a comparative experiment is carried out on the two kinds of data. The experiments in this chapter are divided into four groups: the first group of experiments is to average the data, and four types of exercise effects are selected. The third group of experiments is to use the random forest method to find the characteristics of the significant impact of various types of exercise on the body in the data set; the fourth group of experiments is to use the other two baseline algorithms to find the indicators that various types of exercise have a large impact on the body indicators. Above, four baseline algorithms were used to conduct comparative experiments, and these five methods were compared with the ground-truth data in the dataset to obtain the evaluation results. The experimental evaluation criterion in this paper is the accuracy of top@k, which is defined as the ratio of the algorithm-based body metric impact matching the ground truth of the ground truth. The higher the accuracy, the more effective the algorithm is. The calculation formula for the accuracy rate (Precision) is

(6) $$\begin{array}{c} Precision=\frac{k}{n}\text{,} \end{array}$$

where *K* represents the number of ground-truth affected indicators, and *n* represents the total number of ground-truth selected indicators.

### 5.2. Analysis of Experimental Results

This paper uses the random forest method to rank the feature importance of the effects of sports on physical indicators based on feature gain and finds that compared with modern school sports, and folk sports have a greater impact on some specific indicators.  Figure 9 shows the ranking of the impact of wrestling sports on physical indicators. It can be seen that the most influential are the average grip strength, cardiac function index, one-minute sit-ups, waist circumference, standing rotation, 50 m sprint, and back muscle strength. Wrestling sports mainly exercise strength, and the experimental results are in line with our cognition.

Figure 10 shows the rank of impacts of podiatric sports on physical indicators. It can be seen that waist circumference, cardio index, vertical rotation, 50 m sprint, repeated straddling, body weight, and cross change running have the greatest impacts. Competitive foot sports mainly exercise physical function and reaction ability, especially the physical function of the lower body. The experimental results are in line with our cognition.

Figure 11 shows the order of the influence degree of skill sports on physical indicators. It can be seen that waist circumference, cardio index, body rotation in standing position, single-legged standing with eyes closed, 50 M sprint, body weight, repeated straddling, and cross-turn running have the greatest influence. Of the eight indicators with a higher degree of influence, three indicators reflect changes in body function, and five indicators reflect changes in reaction power. Skill sports mainly exercise reaction power, and the experimental results are consistent with our cognition.

Similarly, studies the influence of four types of sports on physical effects by using the random forest to make feature selection, similar to the feature selection of elastic network. Studies have shown that four types of physical activity can actually increase metabolism and improve physical function. It includes improving muscle strength and endurance, stretching muscles and collaterals, stretching bones and joints, exercising waist circumference and vital capacity, and strengthening body coordination and reaction sensitivity. In addition, we can also see that various types of sports have different emphases on the ability to exercise. For example, wrestling sports mainly exercise our upper body function and improve the fitness effect of the upper body, which is reflected in the improvement of grip strength and back muscle strength, etc.; it is reflected in the changes in waist circumference, cardiac function index, upright rotation, 50 m sprint, repeated traverse, body weight, and cross-direction running; skill sports are more inclined to exercise our reflexes and sensitivity, etc., reflected in the changes of 50 m sprint, round-trip running, and other indicators; now, school sports focus on all-round development, suitable for students' development, can strengthen the body, enhance physical fitness, and improve the level of sports skills. At the same time, by using the results obtained by our assessment method, physical education teachers can guide students' physical training accordingly and purposefully exercise students' skills and bodies.

This chapter proposes a research and evaluation of sports effects based on a random forest algorithm. The experimental results obtained by using the method in this chapter are consistent with people's subjective cognition and expert judgment. Compared with the baseline method, this method is a simple and practical way of sports effect evaluation and provides a reference for the development of sports effect evaluation in the future. The comparison with four classical methods in the experiment shows that the method proposed in this chapter has higher classification accuracy and can be applied to the evaluation of sports effects.

## 6. Summary and Outlook

In this paper, we use random forest feature selection to study and evaluate the effect of foot competition. From our research, we can see that sports can speed up metabolism and improve physical function, including promoting muscle power and endurance, stretching muscles and collaterals, running bones and joints, exercise waist circumference, and lung capacity; at the same time, strengthen physical coordination and response sensitivity. In addition, we can also see that various types of sports have different emphases on the ability to exercise. For example, wrestling sports mainly exercise our upper body physical function and improve the fitness effect of the upper body, which is reflected in improving grip strength, back muscle strength, etc.; competition sports tend to be lower body physical indicators exercise, improve running ability, etc., which are reflected in the cardiac index, standing rotation, 50 m sprint, repeated traverse, and cross-direction running, etc.; skill sports tend to exercise reflexes and sensitivity, etc., which are reflected in 50 m sprint, round-trip changes in indicators such as running; now, school sports focus on all-round development, suitable for students' development, and can strengthen the body, enhance physical fitness, and improve the level of sports skills. The majority of young people should always pay attention to physical health, who should not only know the impact of all kinds of sports on the body but also realize that they need to improve their physical health. Through adjustment, construction, and adherence to positive and healthy sports, the right type of sports should be chosen. [4].

## Figures and Tables

**Figure 1:** Research flow chart.

**Figure 2:** Bagging algorithm diagram.

**Figure 3:** Flow chart of random forest algorithm.

**Figure 4:** Changes of adult male physical indexes between 2014 and 2010.

**Figure 5:** Relation between entropy and probability in binomial distribution.

**Figure 6:** Bifurcation diagram of root node based on maximum ratio in dual-class multivalue case.

**Figure 7:** Branch diagram of root node in case of multiple attribute values.

**Figure 8:** Schematic diagram of random forest evaluation algorithm.

**Figure 9:** Ranking of influence degree of wrestling exercises on physical indicators.

**Figure 10:** Rank of influence degree of racepod sports on physical indicators.

**Figure 11:** Ranking of the degree of influence of skill exercises on physical indicators.

## Data Availability

The data used to support the findings of this study are available from the corresponding author upon reasonable request.
